# The combination of red palm oil and rooibos show anti-inflammatory effects in rats

**DOI:** 10.1186/s12950-014-0041-4

**Published:** 2014-12-20

**Authors:** Emma Katengua-Thamahane, Jeanine L Marnewick, Olawale R Ajuwon, Novel N Chegou, Gergő Szűcs, Péter Ferdinandy, Tamás Csont, Csaba Csonka, Jacques Van Rooyen

**Affiliations:** Experimental Antioxidant Research Division, Department of Biomedical Sciences, Faculty of Health and Wellness Sciences, Cape Peninsula University of Technology, Symphony Road, Bellville, Western Cape 7535 South Africa; Oxidative Stress Research Centre, Institute of Biomedical and Microbial Biotechnology, Faculty of Health and Wellness Sciences, Cape Peninsula University of Technology, Symphony Road, Bellville, Western Cape 7535 South Africa; DST/NRF Centre of Excellence for Biomedical Tuberculosis Research and MRC Centre for Molecular and Cellular Biology, Division of Molecular Biology and Human Genetics, Department of Biomedical Sciences, Faculty of Medicine and Health Sciences, University of Stellenbosch, Tygerberg, 7505 South Africa; Department of Biochemistry, University of Szeged, Szeged, Dom ter 9, Szeged, H-6720 Hungary; Pharmahungary Group, Hajnoczy u 6, Szeged, 6722 Hungary

## Abstract

**Background:**

Red palm oil (RPO) and rooibos have been shown to exhibit cardioprotective properties. RPO is rich in essential fatty acids and fat soluble antioxidants while rooibos contains polyphenolic compounds with a unique composition of flavonoids. They exert their biological effects in different cellular compartments. Therefore the combination of these two natural food compounds has the potential to enhance the spectrum of available dietary antioxidants in different cellular compartments, which could result in an enhanced protection against certain pathological conditions such as inflammation.

**Methods:**

Male Wistar rats weighing 150-200 g were supplemented with RPO, rooibos or their combination for 28 days. The Langendorff system and the lipoposaccharide (LPS)-induced inflammatory model were used to establish if RPO and rooibos, when supplemented alone or in combination, will reverse the negative effects of LPS on cardiac function at baseline. The effect of dietary intervention was also investigated on modulation of pro-inflammatory and anti-inflammatory cytokines in plasma and myocardial tissue.

**Results and discussion:**

The LPS resulted in induction of systemic inflammation as evidenced by increased levels of IL-1β in plasma of LPS-treated rats compared to their non-treated control counterparts. Dietary supplementation and LPS treatment did not have an effect on baseline cardiac functional parameters. However, the elevation of IL-1β levels in plasma of LPS-induced rats consuming either RPO or rooibos alone were paralleled with increased levels of the anti-inflammatory cytokine, IL-10. The combination of rooibos and RPO was associated with enhanced endogenous production of myocardial IL-10 in LPS-induced rats.

**Conclusion:**

The results of this study indicate that RPO and rooibos when supplemented individually showed anti-inflammatory effect at systemic level while their combination exhibited an enhanced anti-inflammatory effect in the myocardial tissue. Therefore, the findings in the current study argue that the combination of these two natural food substances could be beneficial in clinically relevant conditions where inflammation plays a role.

## Background

Natural food substances have the potential to alter biological functions of cellular and molecular components’ mechanisms by either enhancing the endogenous antioxidant system or through altering the redox signalling status of the cell [1]. This could be beneficial in pathological conditions where oxidative stress and inflammation play an important role. Previous studies have shown that rooibos and red palm oil (RPO) protected the heart against the detrimental effects of ischaemia/reperfusion injury when supplemented individually to rats [2–7]. Experimental evidence has also shown that RPO has potential anti-hypertensive and hypoglycaemic properties [8]. Recent evidence showed that RPO alone or in combination with rooibos can alleviate oxidant-induced hepatotoxicity in male rats [9].

Red palm oil is a product from the fruits of the oil palm tree, Elaeis guineensis (Family Arecaceae) which has been shown to have protective effects against hypercholesterolemia and atherosclerotic plaque formation, despite being high in saturated fatty acids [10,11]. In addition to the various fatty acids that RPO contains, it is also a rich source of a wide spectrum of different lipid soluble antioxidants such as tocopherols, tocotrienols, carotenoids, lycopene and co-enzyme Q10, among others [12–14]. The health benefits of RPO have been attributed to its unique composition of fatty acids and a high content of natural antioxidants [15,13]. RPO is one of the richest sources of natural vitamin E, especially tocotrienols [16]. Vitamin E has been shown to regulate specific cell signalling pathways independent of its antioxidant properties, therefore some of its beneficial effects have been attributed to its ability to modulate signal transduction pathways [17,18]. There is also credible evidence showing that palm oil vitamin E have potential anti-inflammatory properties [19–22].

Rooibos is a uniquely South African herbal tea made from the leaves and stems of the shrub-like leguminous bush, Aspalathus linearis (Brum.f) Dahlg (Fabaceae, Tribe Crotalarieae). It’s flavonoids are unique in that it contains the C-C linked dihydrochalcone glucoside, aspalathin which is oxidized to the flavanones dihydro-iso-orientin and dihydro-orientin during fermentation, the cyclic dihydrochalcone, aspalalinin, the rare 3-dehydroxy dihydrochalcone glucoside, nothofagin, the C-glycosyl flavones orientin, isoorientin, vitexin, isovitexin, and the flavones hemiphlorin and chrysoeriol, luteolin and luteolin-7-O-glucoside and flavonols quercetin and its O-linked glycosides quercetin-3-robinobioside, hyperoside, isoquercitrin and rutin [23–25]. The health effects of rooibos have been proposed to be mostly attributed to the unique polyphenolic composition and its related antioxidant activities [26–30]. Animal and recent human studies have shown that consumption of rooibos or its phenolic components had positive effects on cardiovascular health and inflammation [31–38]. Studies have shown that rooibos may have potential preventive and therapeutic effects against vascular complications in diabetic rats [39]. Aspalathin, the main and unique polyphenol in rooibos, has been shown to positively modulate glucose homeostasis in type 2 diabetes [30], while the antioxidant activity of rooibos has also been linked to its potential anti-inflammatory and DNA protective effects in a rat colitis model [33].

RPO (fat soluble) and rooibos (water soluble) contain different types of antioxidants which reside and exert their biological effects in different cellular compartments [12,13,24,40]. Therefore, it is tempting to speculate that supplementation with a combination of these two natural food compounds can enhance the spectrum of available dietary antioxidants in different cellular compartments and hence offer a better protection against certain pathological conditions such as inflammation. Accumulating scientific evidence shows that inflammation is the underlying pathological cause for most chronic diseases, including cardiovascular diseases, cancer and rheumatoid arthritis [41–45]. Ischaemic heart disease is the commonest form of cardiovascular disease leading to increased morbidity and mortality [46]. The majority of heart attacks and strokes are caused by rupturing of the atherosclerotic plaque in the arterial wall and the tendency of clot formation, which results from plaque rupture [46,42]. It is now a scientifically accepted fact that inflammation in the lining of the artery is the triggering factor in the pathogenesis of atherosclerosis [42]. It is becoming increasingly evident that the use of non-toxic dietary supplements either alone or in combination with pharmacological agents could present an effective strategy in treatment and prevention of the onset of acute and chronic inflammatory diseases [47–50]. In this respect, Haines and co-workers [47] reported that the combination of different phytonutrients provided a more profound anti-inflammatory effect than individual components acting independently. In another study it has been shown that whole tart cherry extract and specific anthrocyanins contained in the tart cherry exhibited synergistic anti-inflammatory effects with lipitor in reducing LPS-IL-6 induced secretion from adipose stem cells [49]. Dietary intervention with a Jerte Valley cherry-based beverage which is a rich source of anthocyanin pigments and other phenolic compounds has been shown to modulate the balance between the levels of pro and anti-inflammatory cytokines in young and old ringdoves by down-regulating the levels of pro-inflammatory cytokines and up-regulating the levels of anti-inflammatory cytokines [48].

Administration of lipopolysaccharide (LPS) to animals is widely used to study responses to in vivo-induced acute systemic inflammation [51,52]. The inflammatory response forms part of the host innate immune response, which represents the first line of defense against invading pathogens or to injury [53]. The cytokine system forms an integral part of the initial response to microbial agents. Cytokines are also important pathophysiological mediators of cardiovascular pathologies such as atherosclerosis and systemic sepsis-induced cardiac dysfunction [54,55]. The isolated rat heart model and the LPS-induced inflammatory model were used to determine if rooibos and RPO supplementation could protect against the negative effect of LPS-induced inflammation on baseline cardiac function.

## Materials and methods

Animals received humane care in accordance with the Principle of Laboratory Animal Care of the National Society of Medical Research and the Guide for the care and use of Laboratory animals of the National Academy of Sciences (National Institutes of Health Publications no. 80–23, revised 1978). The rats had free access to water or rooibos and rat chow. They were individually caged in an experimental animal facility at a constant room temperature of 27°C and exposed to a twelve-hour artificial day-night cycle. The ethical clearance for this study was granted by the Faculty of Health and Wellness Science’s Research Ethics Committee of the Cape Peninsula University of Technology: Ethics Certificate No (CPUT/HW-REC 2010/A004).

### Experimental model

Male Wistar rats weighing 150–200 g were randomly divided into 8 groups and supplemented with fermented/traditional rooibos, red palm oil (RPO) or their combination for 28 days. The four groups were further subdivided into two groups, either receiving 1) No-LPS or 2) LPS injection. Group 1 which is the NO-LPS group consisted of the control group receiving standard rat chow and water, rooibos group receiving standard rat chow and rooibos, RPO group receiving standard rat chow supplemented with RPO 0.2 mL (7 g/kg diet) daily and water. The RPO concentrate was supplied by Carotino SND BHD (Company no. 69046-T) Malaysia. The composition of RPO consumed by the rats is shown in (Table 1).

**Table 1:** **Composition of Carotino RPO premium consumed by the rats**

**Parameters**	**Specifications**	**Typical**
Fatty acids%	0.1 max	0.058
Moisture and impurities,%	0.1 max	0.03
Iodine Value	48-53	51.2
Slip melting point, c	33-37	36.4
Carotenes, ppm	400 min	420
Tocopherols and Tocotrienols, ppm	400 min	860
Nutritional information		
Amt/serving	Qty per 14 g	Qty per 100 g
Energy	518 kJ	3700 kJ
Protein	0.0 g	0.0 g
Fat, total	14 g	100 g
saturated	7.0 g	50.0 g
Trans	0.0 g	0.0 g
polyunsaturated	1.5 g	11.0 g
monounsaturated	5.5 g	39.0 g
Cholesterol	0.0 g	0.0 g
Carbohydrates	0.0 g	0.0 g
sugars	0.0 g	0.0 g
Sodium	0.0 g	0.0 mg
Carotenes as Vitamin A activity	640 ug	4600 ug
Vitamin E	2.5 mg	18.0 mg
Tocopherols	1.7 mg	12.0 mg
Tocotrienols	4.8 mg	34.0 mg

Certificate of analysis prescribed by Carotino 2010.

www.carotino.com.

The rooibos + RPO group received a combination of rooibos and RPO (without LPS treatment). Group 2 which is the LPS group consisted of the control group receiving standard rat chow and water, rooibos group receiving standard rat chow and rooibos, RPO group receiving standard rat chow supplemented with RPO 0.2 mL (equivalent to 7 g/kg diet) daily and rooibos + RPO group receiving the combination of rooibos and RPO (with LPS treatment). Superior grade fermented rooibos was provided by Rooibos Ltd (Clanwilliam, South Africa). The rooibos aqueous extract was prepared by the addition of 100 ml of freshly boiled water to 10 g of tea leaves, filtered and stored at −40°C, and diluted 5 times, a concentration customarily used for tea consumption purposes, before being given to the rats [56]. Phenolic content, antioxidant capacity and flavonoids composition of the rooibos consumed by the animals are as analyzed by Ajuwon et al. [9]. The animals were given 100 ml of the freshly diluted rooibos every second day. The rooibos and water consumption was monitored throughout the feeding period and there were no statistical differences observed in either rooibos or water consumption among the experimental groups (data not shown). At the end of the feeding period (28 days), 18 hours prior to sacrificing, animals in the LPS group were injected (intraperitoneal) with lipopolysaccharide (Escherichia coli serotype) to induce inflammation. The LPS was dissolved in sterile filtered phosphate buffered saline (PBS) to obtain 0.5 mg/kg body weight in 0.1 ml [51]. The animals in the NO-LPS were injected (intraperitoneal) with 0.1 ml of PBS (Table 2).

**Table 2:** **Study design illustrating the experimental groups and study protocol**

	**NO-LPS**				**LPS**			
**Groups**	**Control**	**Rooibos**	**RPO**	**RB + RPO**	**Control**	**Rooibos**	**RPO**	**RB + RPO**
Feeding time	28 days	28 days	28 days	28 days	28 days	28 days	28 days	28 days
Treatment	PBS	PBS	PBS	PBS	LPS	LPS	LPS	LPS
	*Heart excision and perfusion protocol				*Heart excision and perfusion protocol			

RB: rooibos.

RPO: red palm oil.

LPS: liposaccharide.

Treatment: 0.5 mg/kg LPS was injected intraperitoneally to induce inflammation while 0.1 ml PBS was injected as a vehicle in control groups 18 hours prior to sacrificing.

^*^Hearts were excised and perfused for 20 minutes in a Langendorrf mode, baseline heart function was recorded at 20 minutes after which hearts were freeze clamped for cytokine analysis.

At the end of the feeding period and inflammation injection protocol, rats were fasted for 16 hours before sacrificed and anaesthetized with an intraperitoneal injection of 2 mg/kg intraval sodium (sodium pentobarbital). Blood was collected from the abdominal aorta (approximately 5–8 ml) and placed into plain tubes for cytokine analysis. Serum was then separated immediately by centrifuging at 5000 g for 5 min at 4°C, the samples were then stored at −80°C till analysis were performed. Hearts were rapidly excised and placed in ice-cold Krebs-Henseleit buffer and transferred to the Langendorff perfusion system. Hearts were perfused with a Krebs-Henseleit buffer equilibrated with 95% O_2_ and 5% CO_2_ at 37°C (118.5 mM NaCl; 4.75 mM KCl; 1.2 mM MgCl 6 H_2_O; 1.36 mM CaCl_2_; 25.0 mM NaHCO_3_; 1.2 mM KH_2_PO_4_; 11.0 mM glucose) and a perfusion pressure of 100cmH2O was maintained throughout the protocol. Hearts were mounted to the Langendorff system and perfused for 15 minutes. Coronary flow, heart rate, LVDevP, RPP, ±dp/dt max derivatives, EDLVP were documented at baseline phase. LVDevP was measured with the aid of a balloon made from transparent sandwich wrap film inserted into the left ventricle through the opening of the left atrium. The balloon was connected to a power lab system (AD Instruments Pty Ltd., Castle Hill, Australia). After insertion, the balloon was inflated to 2 mmHg, and the contraction force of the heart against the balloon caused water displacement that was converted to pressure. The systolic and diastolic pressures as well as the heart rate and minimum and maximum derivatives were documented on the computer. At the end of the perfusion protocol hearts were removed from the system and stored at −80°C till biochemical analysis were performed.

### Immunoassay for plasma and myocardial cytokine analysis

Analyses of samples were performed on undiluted myocardial tissue homogenates which were originally prepared in phosphate buffer at a dilution of 1:4. In order to analyze the myocardial cytokines, hearts from all the 8 groups were freeze-clamped with Wollenberger clamp pre-cooled in liquid nitrogen. The heart samples were then grinded into powder and 100 mg of heart tissue powder was diluted with 500 μl of phosphate buffer. The mixture was homogenized by ultrasonic homogenizer at maximum power (2×20 sec), and the homogenate was centrifuged at 4°C for 20 minutes at 5000 g. The supernatant was collected and stored at −80°C till analyses were carried out. Protein tissue content was determined using Bradford technique [57]. Plasma and myocardial IL-1 beta, IL-6 and IL-10 levels were measured using the Bio-Plex bead array system (Bio Rad Laboratories, USA). Assays were carried out in 96-well filter plates, while the rat cytokine kits, (Cat#: RCYTO-80 K) were obtained from Millipore (USA). Samples were evaluated in duplicate. All levels of analytes in quality control reagents included in the kits were within the expected references ranges.

### Data analysis

Results were expressed as mean ± standard error of the mean (SEM). Differences between the NO-LPS control group and the LPS control group were determined using an unpaired Student’s *t*-test. To compare differences in multiple groups, ANOVA followed by FisherLSD post hoc test was used. P < 0.05 was considered to be statistically significant difference.

## Results

### Plasma cytokine levels

#### IL-1 β

The plasma pro-inflammatory cytokine IL-1β was significantly increased (#p < 0.05) in LPS control (positive controls) rats (367.52 ± 60 pg/ml) when compared to the NO-LPS control (negative controls) rats (63.71 ± 10 pg/ml) (Figure 1a). No differences were observed in plasma.

**Figure 1:** **Effects of inflammation, rooibos and RPO on plasma IL-1β (a), IL-6 (b), and IL-10 (c) levels.** Results are means ± SEM, n = 4-8/group. #p < 0.05: LPS control vs NO**-**LPS control, *p < 0.05: treated vs. corresponding control. RPO: Red palm oil.

IL-1β of the rooibos and RPO-supplemented LPS-treated rats compared to the LPS control. No significant differences were observed between RPO alone and the combination treatment compared to the LPS control (Figure 1a).

#### IL-6

The level of plasma pro-inflammatory cytokine, IL-6 in the positive control rats was not significantly different from the levels in the negative control animals. There were also no differences observed in plasma IL-6 of LPS-induced rooibos and RPO-supplemented rats compared to the positive control (Figure 1b).

#### IL-10

The plasma anti-inflammatory cytokine, There were no differences observed in plasma IL-10 levels between the negative control and the positive control, however, a significant increase (*p < 0.05) in plasma IL-10 level observed in LPS-induced rats consuming rooibos (4082.19 ± 180 pg/ml) compared to the positive control (1462.63 ± 372 pg/ml). A similar pattern of results were also observed for LPS-induced rats supplemented with RPO, where the plasma IL-10 level was significantly (*p < 0.05) increased (2375.28 ± 264 pg/ml) compared to the positive control (1462.63 ± 372 pg/ml). There were no differences observed in plasma IL-10 level of the LPS-induced rats consuming the combination of rooibos and RPO compared to the positive control (Figure 1c).

### Myocardial cytokine levels

#### IL-1 β

When considering the myocardial IL-1β levels, there were no differences observed between the NO-LPS control and the LPS control animals. The level of myocardial IL-1β was significantly (*p < 0.05) increased in LPS-induced rats consuming the rooibos (172.36 ± 23 pg/ml) when compared to the LPS control (73.29 ± 14 pg/ml) rats (Figure 2a).

**Figure 2:** **Effects of inflammation, rooibos and RPO on myocardial IL-1β (a), IL-6 (b), and IL-10 (c) levels.** Results are means ± SEM, n = 5-7/group. #p < 0.05: LPS control vs NO**-**LPS control, *p < 0.05: treated vs. corresponding control. RPO: Red palm oil.

#### IL-6

Myocardial IL-6 was significantly (#p < 0.05) lower in the positive control (121.53 ± 23 pg/ml) compared to the negative control (233.85 ± 38 pg/ml) rats. The level of myocardial IL-6 was significantly (*p < 0.05) increased in LPS-treated rats consuming rooibos (235.58 ± 38 pg/ml) compared to the positive control (121.53 ± 23 pg/ml). The LPS-induced rats which consumed the combination of rooibos and RPO also showed a significant (*p < 0.05) increase in myocardial IL-6 (283.50 ± 29 pg/ml) compared to the LPS control (121.53 ± 23 pg/ml), (Figure 2b).

#### IL-10

When considering the myocardial IL-10 levels, significantly (#p < 0.05) increased levels of myocardial IL-10 were measured in the negative control (915.60 ± 71 pg/ml) compared to the positive control (468 ± 60 pg/ml). While the combination of rooibos and RPO significantly (*p < 0.05) increased myocardial IL-10 levels (739.09 ± 48 pg/ml) compared to positive control. The LPS-induced rats consuming either rooibos or RPO alone did not show significant differences in induction of myocardial IL-10 compared to the positive control (Figure 2c).

## Discussion

The aim of the current study was to induce inflammation in vivo and to establish if dietary supplementation with rooibos and RPO would reverse or suppress the effects of inflammation. We have shown that administration of LPS induced systemic inflammation as evidenced by elevated levels of IL-1β, the inflammation marker, in the plasma of LPS-treated animals compared to non-treated animals. Consumption of either rooibos or RPO alone was associated with elevated levels of plasma anti-inflammatory cytokine (IL-10) in the LPS-induced rats. The results indicate a potential anti-inflammatory property of rooibos and RPO at systemic level when supplemented individually. However, the combination of rooibos and RPO significantly enhanced endogenous myocardial IL-10 level in LPS-induced rats, arguing for potential protection against inflammation on organ level.

### Effects of inflammation, rooibos and RPO on IL-1β

The increased levels of plasma IL-1β in the LPS-induced rats indicate that there was induction of inflammation in response to the presence of the endotoxin (LPS), (Figure 1a). IL-1β is one of the initial pro-inflammatory cytokines to be released in response to the invading microbial pathogens (specifically the lipopolysaccharide, an endotoxin embedded within the bacterial membrane) and it plays a crucial role in the induction of inflammation [58]. Therefore, increased levels of circulating IL-1β are indicative of a systemic inflammatory response [59,60]. The response to LPS is initiated upon the recognition of LPS by the LPS-binding protein, following the binding of LPS to its binding protein a series of multiple complex signalling pathways is initiated. This will ultimately result in activation of the Toll-like Receptor (TLR) 4 through various adaptor proteins leading to NF-κB activation and eventual induction of inflammatory cytokines [61–64]. LPS triggers the release of inflammatory cytokines from various cells of the immune system, the released cytokines leads to an acute inflammatory response directed towards the invading pathogen [65–67]. The finding of elevated plasma levels of IL-1β therefore confirms that inflammation was induced in the current model. Our results are in agreement with previous reports by Ohsaki and co-workers [51] which used a similar dose of LPS and showed increased IL-6 mRNA levels indicating that inflammation was induced. Our results also show that supplementation of either rooibos or red palm oil, together and separate, could not prevent an increase in plasma IL-1β.

However, in the myocardium, our results show that consumption of rooibos in the LPS-induced rats was associated with increased myocardial levels of IL-1β compared to the positive control, while RPO and rooibos + RPO did not affect the induction of myocardial IL-1β (Figure 2a). Myocardial and endothelial cells have the capacity to respond to LPS via activation of the TLRs leading to induction of inflammatory cytokines [67]. The role of cytokines in inflammation is complex and is determined by various factors such as the magnitude of cytokine induction, the presence of receptors to cytokines and also by the presence of antagonist mediators such as anti-inflammatory cytokines. The increased levels of myocardial levels of IL-1β in the LPS-induced rats consuming rooibos may represent a normal cellular response to the presence of the endotoxin [68], especially because the observed increases in myocardial levels of IL-1β in LPS-induced rats consuming rooibos were not associated with alterations cardiac function.

### Effects of inflammation, rooibos and RPO on IL-6

Dietary intervention with rooibos, RPO or their combination did not have any effect on plasma IL-6 levels in LPS-treated animals and their non-treated counterparts (Figure 1b). There was differential modulation of myocardial IL-6 by the dietary supplements in the LPS-induced supplemented rats. Consumption of rooibos and that of the combination of rooibos and RPO in LPS-induced rats caused an increased in myocardial IL-6 compared to the positive control level comparative to that of the negative control animals (Figure 2b). Even though IL-6 is classically characterized as a pro-inflammation cytokine, it has been shown to have both pro-inflammatory and anti-inflammatory features [69,70]. IL-6 can evoke an anti-inflammatory environment by inducing the production of anti-inflammatory cytokines, such as IL-10 and IL-1ra in humans [70]. Our results show that the increase in myocardial IL-6 in the LPS-induced rats consuming rooibos and rooibos + RPO was associated with enhanced up-regulation of myocardial IL-10. Therefore the elevation of both IL-6 and IL-10 indicates that in this instance, IL-6 might be acting as an anti-inflammatory cytokine leading to enhancement of IL-10 production. There is evidence showing that in some instances acute elevation of IL-6 may be beneficial, especially following exercise in humans [70]. Xing and co-workers [71] showed that endogenous IL-6 plays an anti-inflammatory role in both local and systemic acute inflammatory responses in mice. This mechanism acts by controlling the level of pro-inflammatory, but not anti-inflammatory, cytokines [72]. Others have also shown that blockade of IL-6 in patients with rheumatoid arthritis led to enhanced cholesterol and plasma glucose levels, indicating a role for IL-6 in modulation of glucose and lipid metabolism [73,74]. Results in the current study would therefore indicate that endogenous IL-6 rather protected than harmed the heart against induction of LPS, especially in the local organ region as is presented in Figure 2b. The results further show that dietary intervention can influence the levels of IL-6 in cardiac tissue. There is also a difference between systemic and local response to IL-6 levels with LPS induction in the presence of dietary supplements such as red palm oil and rooibos. This needs to be further investigated and clarified.

### Effect of inflammation, rooibos and RPO on IL-10

The current results report that plasma IL-10 levels were significantly elevated in the two LPS-treated groups consuming either rooibos or RPO when compared to the LPS control. However, the LPS-induced rats consuming the combination of rooibos and RPO did not show any effect on plasma IL-10 levels indicating that there was no additional benefit on plasma IL-10 levels when rooibos and RPO were given in combination (Figure 1c). The results indicate that dietary supplementation with rooibos and RPO up-regulated the production of IL-10 in response to the presence of inflammation. IL-10 is a potent anti-inflammatory cytokine whose role is to counteract the effects of pro-inflammatory mediators in various forms of shock and inflammation [75]. Inflammatory cells in the circulation are activated in response to invasion of LPS and the initial induction of inflammatory cytokines in response to LPS is aimed at clearing local effect of the invading pathogen [76]. However, the body has also evolved regulatory systems to maintain the balance between the levels of pro-inflammatory mediators and anti-inflammatory mediators in order to sustain cellular homeostasis and immune system integrity. We have shown that rooibos and RPO, when supplemented individually, enhanced production of IL-10 in the blood, suggesting a potential anti-inflammatory effect at systemic level. Therefore the concomitant release of IL-1 β and IL-10 in plasma of LPS-induced rats consuming rooibos and RPO indicate that dietary intervention with rooibos and RPO modulated the inflammatory response in the model of inflammation by enhancing systemic production of the anti-inflammatory cytokine. Rooibos is rich in various polyphenolic compounds, some unique to the plant as well, of which flavonoids are the most predominant [77]. Various polyphenolic molecules have been shown to exhibit anti-inflammatory activity [78,79]. Polyphenols have a wide range of biological effects which include antioxidant and anti-inflammatory effects [80–83]. In the current study we have shown that rooibos consumption was associated with increased levels of plasma IL-10. This is in line with previous studies where polyphenols were associated with enhanced production of IL-10 and suppression of IL-1β [81].

Just as polyphenols form a vital part of a healthy diet, vitamins are also equally essential for human health. RPO is rich in various forms of vitamin E and carotenoids which function as cellular antioxidants [84,13]. Inflammation and oxidative stress are closely related and are usually common features underlying etiological and pathological mechanisms for most chronic diseases including cardiovascular diseases [85,86]. Both tocotrienols and tocopherol are potent antioxidants and have also been shown to possess potential anti-inflammatory properties [19,22].

Dietary supplementation with the combination of rooibos and RPO resulted in increased myocardial levels of IL-10 in the LPS-induced rats compared to the positive control while, when supplemented individually, rooibos and RPO in the presence of LPS, did not have any effect on myocardial IL-10 levels (Figure 2c), this result could be indicative of a threshold needed to exert the effect, i.e. that of increased IL-10 levels. To our knowledge this is the first evidence showing that the combination of rooibos and RPO resulted in up-regulation of myocardial IL-10 levels. Elevated myocardial levels of IL-10 have been linked to cardio-protection [87]. Endogenous production of IL-10 has been shown to play an important role in maintaining myocardial integrity during ischaemia-reperfusion via modulation of the inflammation response. In this regard Yang et al. [88], reported that genetic deletion of IL-10 was associated with enhanced inflammation and increased myocardial infarction and necrosis.

### Effects of inflammation, rooibos and RPO on baseline cardiac functional parameters

LPS treatment and dietary supplementation with rooibos and RPO did not have an effect on baseline cardiac functional parameters. The increases in plasma IL 1β levels and in myocardial tissue of the LPS-induced rooibos group were not associated with ventricular dysfunction or reduction in coronary flow (Table 3). This is contrary to reports that IL-1β has a negative inotropic effect and that it also leads to endothelial dysfunction [89,54]. The reason for this could be that the dose of LPS that we used in this study was sufficient to induce inflammation but not high enough to induce cardiac dysfunction. In previous studies where ventricular dysfunction was reported, higher doses of LPS were used [90,91]. Lew et al. [92], also reported that sub-lethal dose of LPS had minimal effect on cardiac function. Another plausible reason could be that low doses or sub-lethal doses of LPS have been shown to have a pre-conditioning effect [93–95].

**Table 3:** **Effects of inflammation, rooibos and RPO on baseline cardiac functional parameters in the NO-LPS group and the LPS group**

	**LPS**				**NO-LPS**			
	**Control**	**Rooibos**	**RPO**	**RB + RPO**	**Control**	**Rooibos**	**RPO**	**RB + RPO**
CF (ml/min)	13.92 ± 1.00	13.84 ± 1.00	14.6 ± 1.00	15.2 ± 1.00	14.30 ± 0.60	13.70 ± 0.70	14.60 ± 0.70	15.10 ± 0.20
HR bpm (1/min)	294.33 ± 6.00	277.87 ± 13.00	279.69 ± 15.00	296.313 ± 8.00	293.14 ± 14.00	302.39 ± 12.00	296.86 ± 10.00	300.00 ± 13.00
LVDevP (mmHg)	92.804 ± 6.00	86.40 ± 6.00	86.47 ± 5.00	97.00 ± 3.00	106.25 ± 4.30	89.60 ± 2.40	95.500 ± 4.50	100.90 ± 4.410
RPP (Bpm*mmHg)	27593.83 ± 1814.00	23706.98 ± 660.00	24383.99 ± 2503.00	28319.93 ± 764.00	30133.51 ± 1394.00	24805.68 ± 1366.00	24701.52 ± 1551.00	26176.72 ± 1212.00
dp/dt (+) (mmHg/sec)	2822.951 ± 149.00	2829.72 ± 84.00	2661.67 ± 198.00	2664.75 ± 112.00	3065.48 ± 103.00	2888.66 ± 129.00	2885.71 ± 80.00	2814.45 ± 113.00
dp/dt (−) (mmHg/sec)	1933.91 ± 70.00	1906.73 ± 82.00	1918.94 ± 103.00	1996.27 ± 94.00	2140.53 ± 90.00	1969.86 ± 69.00	2024.86 ± 120.00	1952.45 ± 51.00
EDLVP (mmHg)	10.256 ± 0.92	13.424 ± 2.20	11.558 ± 0.72	12.29 ± 1.34	13.74 ± 2.36	12.93 ± 1.33	12.22 ± 2.24	11.78 ± 1.16
HW (g)	1.17 ± 0.09	1.16 ± 0.05	1.11 ± 0.041	1.09 ± 0.03	1.32 ± 1.0	1.11 ± 0.0	2.82 ± 1.4	1.28 ± 0.1
BW (g)	333.70 ± 4.53	343.90 ± 10.02	346.60 ± 6.80	348.20 ± 3.40	350.20 ± 7.5	352.40 ± 7.4	334.20 ± 8.8	340.40 ± 90

No significant differences were observed in baseline cardiac function between the groups. Results are expressed as SEM, n = 5-7. CF- Coronary flow, HR- Heart rate, LVDevP- Left ventricular developed pressure, RPP- Rate pressure product, dp/dt (+) - maximum of LVDevP derivative, dp/dt (-) - minimum of LVDevP derivative, EDLVP- End diastolic left ventricular pressure, HW- Heart weight, BW- Body weight.

## Conclusion

In this study we have shown that the model that we used to induce inflammation has worked, as evidenced by increased levels of IL-1β in the blood. Evidence presented here, show for the first time, that the dietary combination of rooibos and RPO significantly enhanced the up-regulation of endogenous myocardial anti-inflammatory IL-10 levels, a phenomenon shown to have great potential in cardio-protection. This study also showed that IL-6 in this model acted more like an anti-inflammatory rather than pro-inflammatory mediator. It was also evident from the results that there is a difference in response to LPS injection between the myocardium and the systemic circulation. Therefore, the results argue that the combination of these two natural food substances exhibit potential anti-inflammatory properties worth investigating further.
